The article "Analyzing the tourism efficiency and its influencing factors of China’s coastal provinces" was published in 2024. Journal: PLoS One.

# Analyzing the tourism efficiency and its influencing factors of China’s coastal provinces

**DOI:** 10.1371/journal.pone.0299772

**Published:** 2024-05-17

**Authors:** Changping Yang, Yongxing Xia, Johnny F. I. Lam, Hongxi Chen, Huangxin Chen

**Affiliations:** 1 School of Economics, Fujian Normal University, Fuzhou, China; 2 Faculty of Humanities and Social Sciences, Macao Polytechnic University, Macao, P R China; 3 International College, Ulaanbaatar Erdem University, Ulaanbaatar, Mongolia; Abdelmalek Essaadi University: Universite Abdelmalek Essaadi, MOROCCO

## Abstract

Tourism efficiency has become an important role in promoting tourism competitiveness and driving sustainable development. It is particularly important to identify and agnalyze the factors and mechanisms that affect efficiency. This paper firstly evaluates the tourism efficiency of 11 coastal provinces regions in China from 2010 to 2020 by using the DEA-BBC model that includes undesirable outputs. After that, it investigates the internal driving mechanism of the efficiency change through the Malmquist index and its decomposition. Finally, it analyzes the external influencing elements of tourist efficiency by the Tobit model. The results show that: (1) Although the average value of the tourism efficiency was changed from 0.727 to 0.707, it does not achieve the target. Its trend shows fluctuating from 2010–2020, which indicates that the tourism efficiency of most provincial regions is not optimal. The main factor that restricts tourism efficiency is scale efficiency. (2) By analyzing the dynamic trend, it is found that the average increase of technical efficiency is 14.0%, the average increase of technical change is 9.5%, and the average increase of MI index is 25.4%. It indicates that the overall tourism efficiency of 11 coastal provinces region in China is on the rise. (3) The spatial difference of tourism efficiency is significant, but there is no obvious spatial correlation. (4) The influencing factors of tourism efficiency are consumer demand, industrial structure, labor force and urbanization.

## 1. Introduction

Tourism, a general term for enterprises and institutions that provide services for tourists or various activities related to tourists, plays an important role in promoting the economy. As we know, with the gradual progress of reform and opening, Chinese living standard has been significantly improved, and the tourism demand is constantly growing. The tourism industry has also been significantly developed. Now, China has become the largest tourism market in the world. The rapid economy and social development are benefited from tourism as a pillar industry. The tourism industry already accounted for 10% of China’s GDP. In 2019, the number of Chinese tourists exceeded 6 billion and the total tourism revenue exceeded 6 trillion yuan. It has also been suggested to increase the contribution of tourism to the economic development and quality of resident life [1]. We can see that tourism efficiency has received more attention with the upgrading of tourism. Tourism, as a modern service industry, has interactivity and influence on natural geographical and cultural resources. Therefore, more and more provinces generally focus on tourism efficiency and take advantage of their natural and cultural resources through promoting investment, transportation and star-related hotels. It has formed an extensive growth dominated by scale expansion.

The article "Analyzing the tourism efficiency and its influencing factors of China’s coastal provinces" was published in 2024. Journal: PLoS One.

The sample includes Liaoning, Hebei, Tianjin, Shandong, Jiangsu, Shanghai, Zhejiang, Fujian, Guangdong, Guangxi, and Hainan. The tourism development status of 11 coastal provinces regions in 2020 is shown in Table 1. It uses five indicators to measure the development status: the number of tourists (10,000 people), the number of star-rated hotels, the number of A-level scenic spots, the number of travel agencies, and tourism revenue (100 million yuan).

**Table 1:** Tourism development status of 11 coastal provinces regions in 2020.

Areas	Tourist	Star-rated Hotels	A-level Scenic Spots	Travel Agencies	Tourism Revenue
Fujian	36981.1	279	401	1270	4927.7
Guangdong	23059.5	613	486	3425	4690.6
Guangxi	66092.0	444	611	881	7262.1
Hainan	6455.1	96	69	601	872.9
Hebei	37952.5	285	465	1531	37952.5
Jiangsu	47174.1	399	615	3066	8136.3
Liaoning	30150.0	312	571	1539	2712.2
Shandong	57669.6	539	1227	2685	6019.7
Shanghai	23606.0	188	130	1808	2809.1
Tianjin	14100.0	69	96	516	1354.5
Zhejiang	56978.0	599	827	2885	8264.0

In China, when evaluating tourism efficiency, they always take all regions as a whole, or focus on a specific province. These are unfavorable development levels and uneven growth among regions. This research ignores the difference in development among regions, resulting in certain bias in the conclusions. As the most important economic regions, the GDP of these 11 coastal provinces region accounts for more than half of total GDP in China and it also leads to the development of the national economy. The tourism economy in these 11 coastal provinces region has been growing from 1978, based on excellent tourism resources and infrastructure. In view of the rapid economic growth, the provinces have adopted various measures to enhance their tourism competitiveness which relies on capital and labor input. Tourism also attracts more tourists, brings objective incomes which have reached 9.39 trillion yuan in 2019 and accounted for 22.18% of the total GDP. Even under the influence of the COVID-19, the tourism income also exceeds 10% of the total regional GDP. As developed regions, the transformation, upgrading, quality and efficiency improvement become critical factors to promote 11 coastal provinces’ tourism. But few researchers pay attention to tourism-developed areas. Most of the studies have only analysed phenomena and do not explore the cause. Even if some scholars do research on this, it is based on data from many years ago, and the research results are not timely. Comprehensive and effective measurement of tourism efficiency and exploration of strategies to improve tourism efficiency contribute much to facilitate the transformation of its development mode. The innovation of this paper is to focus on the tourism efficiency in these 11 coastal provinces region of China, with the highest level of tourism economy. By comparing the values from 2010 to 2020, this paper studying in 11 coastal provinces region shows the trends in tourism, to help people get a better understanding of the true picture of China’s tourism.

The article "Analyzing the tourism efficiency and its influencing factors of China’s coastal provinces" was published in 2024. Journal: PLoS One.

The main issues to be resolved in this paper include: (1) Constructing a provincial-level regional tourism efficiency evaluation index system to fully reflect the input and output of China’s tourism industry and the main influencing factors; (2) Revealing the present situation of tourism development in different parts of China and analyzing the influence of external environmental factors on tourism efficiency by determining the tourism efficiency of 11 coastal provinces regions in China from 2010 to 2020; (3) Studying tourism efficiency in these provincial regions. We can not only understand the allocation of tourism resources, but also understand how to utilize resource allocation to promote tourism’s development and expand the scale. Moreover, we can further and better understand the entire Chinese economy.

## 2. Literature review

As an economic phenomenon, tourism efficiency means that the inputs will bring a certain output in periods. The results are used to evaluate the sustainability of tourism. When the input is stable, the higher efficiency means the more output. The tourism efficiency of other famous tourist countries is often discussed. Many scholars pay more attention to tourism efficiency, focusing on travel agencies [2–4], tourist hotels [5–7], and tourist attractions [8, 9]. For example, R and Widodo [10] discussed that the knowledge quality had positive influence on tourism’s competitive advantage. Morrison and Buhalis [11] provided insights on the differences among domestic and foreign markets, acknowledged that the supply sub-sectors of tourism were diverse and highlighted the variations by geographic regions. With a focus on the Indian subcontinent, Chowdhary and Prakash [12] explored various frameworks in relation to the tourism and hospitality industry. Álvaro, Quintero and Carol [13] discussed that heritage and tourism were strongly related to each other. Heritage gave rise to tourist attractions and activities, and tourism enhanced the designation of heritage sites. Todd and E [14] explored the daily experiences of local tourism workers in the expansion of the tourism industry. Gutberlet [15] explored the socio-cultural, economic, and spatial challenges faced in tourism development. Fuarros, Paiva and Calvo [16] took some examples such as a traditional Italian marketplace, a jungle park in Kuala Lumpur, a slum in the Colombian city of Medellín, or the "sun and sand" tourism destinations in Southern Spain, in order to affirm the significance of culture ambiance for tourist consumption. Koščak and O’Rourke [17] explained how the recent global events impacted on local tourism, such as the Covid-19 health crisis and the war in Ukraine. Raana [18] proposed and expounded a structural model that depicted the tripartite relationships among sense of place, attractions and satisfaction by using the data of experiences of a sample of 396 foreign tourists in Shiraz city, Iran. It showed the importance of tourist experiences in boosting the tourism industry and the importance of the attractions on tourist satisfaction. With the persistence of low labor productivity in tourism, Kim, Williams, Park and Chen [19] discussed that there was an urgent need to increase spatial spillover effects of agglomeration economies. Cuffy, Bakas and Coetzee [20] expounded how attractions, music festivals, events and wanderlust affected the tourism industry. Chaabouni [21] used DEA-model to investigate the tourism efficiency in China. The results showed that the tourism efficiency in China was low. At the regional level, the average tourism efficiency in east China was higher than central and west.

The article "Analyzing the tourism efficiency and its influencing factors of China’s coastal provinces" was published in 2024. Journal: PLoS One.

In China, Xing Fumin [22], Wang Zhaofeng [23], Deng [24] and other scholars focus their research on one certain province. For example, Dan, Xianzong, Fayyaz, Nabila and Zulqarnain [25] valued the tourism efficiency of Gansu Province, and then investigated the internal driving mechanism of the efficiency change. Wenhua [26] conducted some research on the tourism efficiency in Guangxi. The results showed that the improvement of technological progress was the most effective way to promote the efficiency growth of tourism in Guangxi. Yaobin, Meizhen, Kongming and Jinhang [27] analyzed the relationships between tourism efficiency and transport. It showed improving the spatial match of tourism efficiency and transport could enhance the sustainability of tourism development. While for other scholars, Dandan [28], Lu Xiaojing and etc [29], paid more attention to the dynamic changes of tourism efficiency in some regions of China. For example, Songsong, Tai and Jianchao [30] took the Yangtze River as a case to analyze the evolutionary process of regional tourism efficiency. Bin, Li and Li [31] measured the environmental pollution and tourism efficiency. It revealed the spatial difference between regional tourism efficiency and tourism scale was obvious, so environmental problems were raised. On the national level, some scholars such as Rui [32], Fang Yelin [33], Zifang, Jiaqi and Weiwei [34] and Yan, Yeqin [35] analyzed the tourism efficiency values of the whole 31 and cities in China from different perspectives. For example, Junli, Chaofeng and Sihan [36] used SBM-DEA model to measure the tourism efficiency of 30 provinces and analyzed the factors and mechanisms that affected efficiency. Zhiliang et al [37] discussed spatial–temporal heterogeneity and the related influencing factors of tourism efficiency in China. The results revealed that low-efficiency regions were mainly concentrated in northern China, while high-efficiency regions were concentrated in southern China. Zhaofeng, Qingfang, Jianhui and Yousuke [38] explored the evolution characteristics of the spatial network structure of tourism efficiency in China at the provincial level from the years 2011–2016.

To sum up, most scholars can use quantitative methods such as DEA model to estimate tourism efficiency. They do not only focus on a certain province, but also on a region or even the whole country. However, few scholars pay attention to the tourism efficiency of coastal areas. At present, there is not a complete and universal evaluation system in China. Combined with the views of the above scholars, this paper takes 11 coastal provincial regions in China as the research cases, uses DEA model to calculate their tourism efficiencies, and innovates the evaluation system of tourism efficiency to make it more in line with the goal of sustainable tourism development in China’s tourism industry.

## 3. Research design

### 3.1 Methodology

#### 3.1.1 DEA-BBC model

Above all, scholars mainly use the DEA model to evaluate the tourism efficiency. DEA model, an important method to evaluate tourism efficiency at present [39], is an efficiency measurement method proposed by Charnes, Cooper, and Rhodes [40] in the 1970s. It is a linear programming model obtained by relevant theories of operational research under the assumption that the return to scale remains unchanged. In 1984, Banker et al. [41] proposed an efficiency measurement model with variable returns to scale, the BBC model, which decomposed the overall efficiency in the CCR model into pure technical efficiency and scale efficiency.

The article "Analyzing the tourism efficiency and its influencing factors of China’s coastal provinces" was published in 2024. Journal: PLoS One.

The DEA model is subdivided into input and output. Input-oriented refers to minimizing the required input variables and maximizing the output by controlling the weight coefficient of input variables under the given conditions of output. It is a non-parametric analysis method based on mathematical programming models. The characteristic is that decision making units can evaluate multi-input and multi-output indicators without estimating and testing parameters, so its conclusion has strong objectivity and scientific. DEA models are adopted in such as: Gu Jiang’s Appraisal and Model Foundation of the Efficiency in Tourism Production in China [42], and Liang Mingzhu’s An Evaluation and Analysis of Tourism Efficiency in Different Cities and Regions of Guangdong Province [43].

In summary, tourism is highly interconnected. Its development is susceptible to various factors and is characterized by volatility. Therefore, the efficiency of the tourism industry is inevitably a dynamic process of changes. Based on the uncertainty of input and output in the tourism, this paper selects an input-oriented DEA-BBC model to measure the economic efficiency of tourism in 11 coastal provinces regions of China. The DEA-BBC model [44] is as follows:

$$\begin{array}{l} \min\theta \\ s.t.\sum_{i=1}^{n}\lambda_{i}X_{i}+S^{-}=\theta X_{i}\\ \sum_{i=1}^{n}\lambda_{i}Y_{i}+S^{+}=Y_{i}\\ \sum_{i=1}^{n}\lambda_{i}=1\\ \lambda_{i},S^{-},S^{+}\geq 0 \end{array}$$ (1)

The results indicate the technical efficiency (TE), pure technical efficiency (PTE) and scale efficiency (SE). The relation between TE, PTE and SE is TE = PTE*SE. When TE = 1, if and only if PTE = 1& SE = 1, it indicates tourism is effective.

#### 3.1.2 Malmquist index

Malmquist index model is a quantitative index to analyze productivity changes in two different periods. This paper uses the Malmquist index model for analysis in order to investigate the changes of tourism industry productivity in a certain period. The Malmqusit model [45] is as follows:

$$TFP=M(y_{t+1},x_{t+1})=\frac{d^{t+1}(x_{t+1},y_{t+1})}{d^{t}(x_{t},y_{t})}{\left[\frac{d^{t}(x_{t+1},y_{t+1})}{d^{t+1}(x_{t+1},y_{t+1})}*\frac{d^{t}(x_{t},y_{t})}{d^{t+1}(x_{t},y^{t})}\right]}^{\frac{1}{2}}$$ (2)

The TFP index from T period to T+1, is the change index of productivity. When TFP>1, it means that the productivity is increasing. When TFP<1, it means that the productivity is decreasing. When TFP = 1, it means that the productivity remains unchanged. TFP is decomposed into technical efficiency change index (TEC) and technical progress change index (TC), and TFP = EC*TC. It will help us to understand the relationship between various changes. When TEC>1, it indicates an improvement in relative technical efficiency and that a certain region is closer to the production frontier. When TC>1, it indicates progress in production technology. TEC can be further decomposed into scale efficiency change (SEC) and pure technical efficiency change (PTEC). If PTEC or SEC is greater than 1, it means that it has a positive effect on tourism efficiency.

The article "Analyzing the tourism efficiency and its influencing factors of China’s coastal provinces" was published in 2024. Journal: PLoS One.

#### 3.1.3 Coordination model

Sustainable development of tourism is based on sustainable development of the economy. Coordination model is a quantitative indicator that measures the degree of coordination among various elements within a system [46]. This paper uses it to measure whether the macroeconomy and tourism are coordinated or not in order to demonstrate tourism efficiency in the region. The expression [47] is as follows:

$$C=\sqrt{\frac{{\left[4*f(x)g(x)\right]}^{2}}{{\left[f(x)+g(x)\right]}^{4}}*\frac{f(x)+g(x)}{2}}$$ (3)

C ranges from 0 to 1. If the result is closer to 1, it indicates that tourism is more coordinated with the macroeconomy, and tourism is more sustainable. When C = 1, it means tourism is fully in line with the macroeconomy.

#### 3.1.4 Tobit model

This paper analyzes the relevant factors affecting tourism efficiency, including consumer demand, industrial structure, labor force, urbanization and fixed asset investment. The parameter estimation obtained by using the Tobit model has the characteristics of unbiased and consistency in this paper. The Tobit model was proposed by James Tobit, and this model is mainly adapted to the situation when the dependent variable is partially continuously distributed and partially discrete. The Tobit model [48] is as follows:

$$y_{i}=\beta_{0}+\beta_{1}x_{1i}+\beta_{2}x_{2i}+\beta_{3}x_{3i}+\beta_{4}x_{4i}+\beta_{5}x_{5i}+\varepsilon_{i}$$ (4)

In the expression, β is the unknown parameter estimator vector, x_i_ is the explanatory vector and y_i_ represents the tourism efficiency, which measured by DEA are [0,1]. And ε is the random error term.

### 3.2 Input-output variables

The DMUs need to have inputs in order to obtain corresponding outputs. Labor, capital and land are considered as the main driving force for economic growth. Compared with the primary and secondary industries, tourism is less dependent on land. So, scholars do not consider land factors when studying tourism efficiency. LSY Han estimates the use and preservation values of natural and/or cultural resources in five distinctive national parks. The empirical results show that natural and/or cultural resources of the sample national parks possessed considerable use and preservation values [49]. Michaela Stanickova, K Skokan used part of the Country Competitiveness Index (CCI) to competitiveness evaluation as input variables to analyse a degree of efficiency in Austria and Germany [50]. Hospitality is one of the key sectors in tourism. In order to attract customers, hotels must be competitive, so Aurélie Corne measures hospitality efficiency as an important aspect of tourism research [51]. Tourism expenses, number of employees and number of beds are used as input variables; tourism receipts, tourist arrivals and number of nights spent are used as output variables in HS Kurt’s study [52]. I Ili&I Petrevska used tourism expenses and the number of beds as input parameters, while using the number of arrivals, the number of nights spent and tourism revenue in 2016 as output parameters in order to determine tourism efficiency of Serbia and the surrounding countries [53]. Z Wang, S Xu take labor, assets, attraction of tourism resources and transport as the input indicator while arrivals of tourists and income of tourism as the output indicator to evaluate tourism efficiency in Zhangjiajie, China [54]. Fei Lu, HuaiGuo Ren take the number of direct working people, the attractiveness of the cultural tourism industry, technological progress and energy consumption as the input indicator while the added value of cultural industry and tourism revenue as the output indicator to evaluate the culture and tourism integration efficiency [55]. Moaaz Kabil used the length of shoreline, area, investments, quality of coral reefs, hotels number and accommodation capacity as input parameter, while using the employees numbers and tourist numbers as output parameter to estimate the efficiency of tourism centers in the Egyptian Southern Red Sea region for applying the blue economy conceptual kernel [56].

The article "Analyzing the tourism efficiency and its influencing factors of China’s coastal provinces" was published in 2024. Journal: PLoS One.

So, this paper also chooses input factors from the perspective of labor, capital and resources. Drawing on the previous research results, this paper innovatively chooses macro indicators to evaluate these three factors, so as to reflect the macro efficiency, among which: (1) The number of people employed [52] in the tourism industry is taken as labor vector. The fixed assets of the tourism industry [54] and passenger volume [57] are on behalf of capital. As for tourism resources richness, we give A-level scenic spots [49], star-rated hotel [57] and travel agencies [53] respectively, multiplied by the corresponding number. Above all is taken as input vectors. Total income of tourism and the number of tourists [54] are taken as output vectors. Based on the input-output theory, an evaluation index system for tourism efficiency in various provincial regions is constructed from the angle of economy and human utilization (shown as Table 2).

**Table 2:** Evaluation index system for tourism efficiency in 11 coastal provinces regions.

First-level index	Second-level index	Third-level index	Reference source
Input index	Resource	Number of A-level scenic spots	Literature (Lee & Han, 2002) [49]
		Number of star-rated hotels	Literature (Corne, 2015) [51]
		Number of travel agencies	Literature (Ilić & Petrevska, 2018) [53]
	Capital	Fixed assets of Tourism Industry	Literature (Xu, 2018) [54]
		Passenger volume	Literature (Aissa & Goaied, 2016) [57]
	Labor	Number of employees in Tourism-related industries	Literature (Soysal-Kurt, 2017) [52]
Output index	Revenue	Total income of tourism	Literature (Xu, 2018) [54]
	Tourist	Number of tourists	Literature (Xu, 2018) [54]

Any slight change in either the source or the host destination can have a large impact on tourism demand, and the impact of major emergencies on the tourism industry is even more self-evident [58]. The outbreak of the COVID-19 has hit the pause button for the tourism industry. The three-year-long outbreak has also had a huge impact on tourism, adding to the uncertainty of the Chinese economy in transition. The tourism efficiency cannot be truly reflected. So, this paper uses the data for 2010–2020 as input-output variables. The data for each indicator are all official data from 2010–2020, the National Bureau of Statistics of China (http://www.stats.gov.cn/).

## 4. Analysis of the empirical results

### 4.1 DEA analysis

This paper calculates the tourism efficiency of 11 coastal provinces regions in China by using DEAP2.1 software (shown as Table 3).

**Table 3:** Tourism efficiency and decomposition for 11 coastal provinces regions.

Year	Proj.	Fujian	Guangdong	Guangxi	Hainan	Hebei	Jiangsu	Liaoning	Shandong	Shanghai	Tianjin	Zhejiang
2010	TE	0.868	1.000	0.672	0.672	0.330	0.667	1.000	0.960	0.499	0.632	0.697
	PTE	1.000	1.000	1.000	1.000	1.000	1.000	1.000	1.000	1.000	1.000	1.000
	SE	0.868	1.000	0.672	0.672	0.330	0.667	1.000	0.960	0.499	0.632	0.697
		irs	-	irs	irs	irs	irs	-	irs	irs	irs	irs
2011	TE	0.921	1.000	0.673	0.673	0.433	0.699	0.791	0.936	0.991	0.649	0.726
	PTE	1.000	1.000	0.983	0.983	1.000	1.000	1.000	1.000	1.000	1.000	1.000
	SE	0.921	1.000	0.684	0.684	0.433	0.699	0.791	0.936	0.991	0.649	0.726
		irs	-	irs	irs	irs	irs	irs	irs	irs	irs	irs
2012	TE	0.930	1.000	0.671	0.671	0.421	0.740	0.900	1.000	1.000	0.543	0.736
	PTE	1.000	1.000	1.000	1.000	1.000	1.000	1.000	1.000	1.000	0.977	1.000
	SE	0.930	1.000	0.671	0.671	0.421	0.740	0.900	1.000	1.000	0.556	0.736
		irs	-	irs	irs	irs	irs	irs	-	-	irs	irs
2013	TE	1.000	0.995	0.742	0.742	0.487	0.788	0.908	1.000	0.919	0.734	0.785
	PTE	1.000	0.997	1.000	1.000	0.997	1.000	1.000	1.000	0.987	0.974	1.000
	SE	1.000	0.999	0.742	0.742	0.489	0.788	0.908	1.000	0.931	0.753	0.785
		-	drs	irs	irs	irs	irs	irs	-	irs	irs	irs
2014	TE	0.879	0.992	0.754	0.754	0.563	0.855	1.000	0.967	0.937	0.762	0.681
	PTE	0.984	1.000	0.990	0.990	1.000	1.000	1.000	1.000	0.993	0.974	0.978
	SE	0.894	0.992	0.762	0.762	0.563	0.855	1.000	0.967	0.943	0.782	0.697
		irs	irs	irs	irs	irs	irs	-	irs	irs	irs	irs
2015	TE	0.882	0.998	0.695	0.695	0.651	0.894	0.852	0.917	0.787	0.867	1.000
	PTE	0.985	1.000	0.945	0.945	1.000	1.000	0.934	1.000	1.000	0.992	1.000
	SE	0.896	0.998	0.736	0.736	0.651	0.894	0.912	0.917	0.787	0.874	1.000
		irs	irs	irs	irs	irs	irs	irs	irs	irs	irs	-
2016	TE	0.981	1.000	1.000	1.000	0.755	0.926	1.000	0.926	0.980	0.924	1.000
	PTE	0.998	1.000	1.000	1.000	1.000	1.000	1.000	1.000	1.000	1.000	1.000
	SE	0.982	1.000	1.000	1.000	0.755	0.926	1.000	0.926	0.980	0.924	1.000
		irs	-	-	-	irs	irs	-	irs	irs	irs	-
2017	TE	0.938	1.000	0.792	0.792	0.837	0.966	0.871	0.959	1.000	0.890	1.000
	PTE	1.000	1.000	0.974	0.974	1.000	1.000	1.000	0.999	1.000	0.980	1.000
	SE	0.938	1.000	0.814	0.814	0.837	0.966	0.871	0.961	1.000	0.908	1.000
		irs	-	irs	irs	irs	irs	irs	irs	-	irs	-
2018	TE	0.970	1.000	0.860	0.860	0.922	0.988	0.972	1.000	1.000	1.000	1.000
	PTE	1.000	1.000	0.996	0.996	1.000	1.000	1.000	1.000	1.000	1.000	1.000
	SE	0.970	1.000	0.863	0.863	0.922	0.988	0.972	1.000	1.000	1.000	1.000
		irs	-	irs	irs	irs	irs	irs	-	-	-	-
2019	TE	1.000	1.000	1.000	1.000	1.000	1.000	1.000	1.000	1.000	1.000	1.000
	PTE	1.000	1.000	1.000	1.000	1.000	1.000	1.000	1.000	1.000	1.000	1.000
	SE	1.000	1.000	1.000	1.000	1.000	1.000	1.000	1.000	1.000	1.000	1.000
		-	-	-	-	-	-	-	-	-	-	-
2020	TE	0.729	0.479	0.804	0.804	0.546	0.707	0.631	0.731	0.716	0.828	0.798
	PTE	1.000	1.000	1.000	1.000	1.000	1.000	1.000	1.000	1.000	1.000	0.965
	SE	0.729	0.479	0.804	0.804	0.546	0.707	0.631	0.731	0.716	0.828	0.826
		irs	irs	irs	irs	irs	irs	irs	irs	irs	irs	irs

The TE of 11 coastal provinces regions in China from 2010 to 2019 is: 0.727, 0.774, 0.784, 0.831, 0.838, 0.855, 0.954, 0.919, 0.926, 1.000. The overall efficiency of tourism in 2010 was effective in only 2 provinces, with an overall average efficiency of 0.727 and the lowest of 0.333 (Hebei). In 2019, overall provincial regions have reached the optimal level. It means the overall tourism efficiency is on the rise, except for the impact of the epidemic in 2020, which led to a decrease in tourists and revenue. Among them, the average TE has reached more than 85% of the optimal level. Though it indicates that the overall tourism efficiency is at a high level, it needs to be improved in the future. And the tourism efficiency of 11 coastal provinces regions is uneven. Guangdong, Shandong and Fujian have reached the optimal level, while Tianjin, Hainan, Guangxi and Hebei are lower than the average. And the “irs” indicates that the efficiency shows an increasing trend from 2010 to 2020. As a result, the tourism efficiency of 11 coastal provinces regions is showing a positive trend, and higher output can be obtained by increasing input. This also shows that tourism is developing as a good target.

The article "Analyzing the tourism efficiency and its influencing factors of China’s coastal provinces" was published in 2024. Journal: PLoS One.

The PTE of 11 coastal provinces regions in China is higher than TE. PTE has all reached the optimal level in most years from 2011 to 2020, and there is no obvious change in the urban pattern. As the regions open to the world, the overall provincial regions easily obtain more on advanced management and technology to promote the development of tourism.

The SE of 11 coastal province regions in China is slightly higher than the TE, while the PTE scatter mostly concentrates on a straight line, indicating that the change trend of the SE is consistent with the change trend of TE. It indicates the SE plays a leading role in the comprehensive efficiency, while PTE plays a supplementary role. There are significant differences among the 11 coastal provinces regions. Southern areas outperform the northern areas, and Hebei is lowest, indicating southern provinces have high utilization of tourism inputs. This is due to the differences in regional development patterns and tourism resources. Regions such as Hebei with a focus on industry are struggling to develop tourism. Hainan lacks cultural resources which are important in tourism. So this tourism does not achieve the optimal output. They need to expand production capacity and invest more human, material and financial resources to develop tourism.

### 4.2 Malmquist analysis

In order to evaluate the change of tourism efficiency accurately in overall provincial regions from 2010 to 2020, this paper applies the Malmquist index model to study the dynamic change trend (shown as Table 4).

**Table 4:** Average Malmquist index and decomposition for 11 coastal provinces regions.

Area	EFFCH	TECHCH	PECH	SECH	MI index
Fujian	1.127	1.082	1.042	1.216	1.370
Guangdong	1.162	1.026	1.132	1.320	1.534
Guangxi	1.090	1.098	0.993	1.000	1.090
Hainan	1.098	1.098	1.000	1.004	1.102
Hebei	1.057	1.077	0.982	0.954	1.009
Jiangsu	1.132	1.051	1.078	1.292	1.463
Liaoning	1.132	1.126	1.006	1.032	1.169
Shandong	1.199	1.057	1.135	1.161	1.392
Shanghai	1.186	1.126	1.053	1.038	1.231
Tianjin	1.232	1.206	1.022	1.003	1.236
Zhejiang	1.112	1.103	1.009	1.082	1.204
Mean	1.140	1.095	1.041	1.100	1.254

As for regional average, the technical efficiency change increased by 14.0%, and technical change increased by 4.8%. Such an increase prompts an increase of 25.4% in the MI index. The results show that the overall tourism operation efficiency of 11 coastal provinces regions has a growing trend. Comparing Tables 1 and 2, it is easy to find that overall regions’ tourism efficiency shows increasing trend, indicating its high input-output efficiency level. It is proved that the tourism of the 11 coastal provinces regions has done relatively well in management and technology.

The article "Analyzing the tourism efficiency and its influencing factors of China’s coastal provinces" was published in 2024. Journal: PLoS One.

Guangdong, Jiangsu and Shandong all performed well, and the MI index ranked the top three among 11 coastal provinces regions, indicating that the tourism industry in these three provinces has achieved a high level in tourism management and development orientation. They have also reached the best level of efficiency in most years, because they enjoy unique advantages in tourism resource allocation. In particularly Guangdong outperforms tourism in other provinces, which takes tourism as the foundation and attracts a large number of high-level tourism talents.

Among them, the pure technical efficiency of Guangxi and Hebei shows a declining trend. This indicates these provinces have low input-output efficiency level. Hebei emphasizes industrial development over tourism investment, which makes up Hebei’s flaws in tourism technical efficiency. The tourism operation efficiency of Hebei is the worst, and the pure technical efficiency is only 0.982, which is at the lowest level in 11 coastal provinces regions. The reason why the MI of Guangxi is too low lies in the insufficient change of scale efficiency. Compared to other regions, Guangxi is in the central part of China, whose economy is underdeveloped. It relies on extensive growth, resulting in excessive waste of tourism. Its growth trend shows as V-shaped, indicating its tourism is not stable, and its development is greatly influenced by internal or external factors.

Overall, if Hebei or Guangxi wants to achieve higher output, it could not only improve resource utilization efficiency, but also need to maintain to bring its tourism operation scale back to the right track. Meanwhile, they also need to pay more attention to improving the management and technology.

### 4.3 Differences in tourism of 11 coastal provinces regions

In order to understand the trend of tourism efficiency among 11 coastal provinces regions in China, this paper selected the DEA data in 2010, 2015 and 2020, using ArcGIS 10.5 software to describe the time evolution of tourism in 11 coastal provinces. According to the rules, it is divided into 5 intervals: lowest, low, average, high, highest. The results are shown in Figs 1–3:

**Fig 1:** Time evolution of DEA in 11 coastal provinces regions from 2010.

The article "Analyzing the tourism efficiency and its influencing factors of China’s coastal provinces" was published in 2024. Journal: PLoS One.

**Fig 2:** Time evolution of DEA in 11 coastal provinces regions from 2015.

**Fig 3:** Time evolution of DEA in 11 coastal provinces regions from 2020.

According to Figs 1–3, the tourism efficiency of 11 coast provinces regions is varied in the period:

1. In 2010, there were large differences among 11 provinces regions, and Guangdong, Shandong, and Liaoning had best value. With abundant resources and effective investment, they stand out.
2. In 2015, Guangdong, Shandong and Liaoning were still ahead of the rest of the regions. In contrast, other regions had reduced tourism efficiency due to excessive investment, especially in Jiangsu, Fujian and Zhejiang. The difference in tourism efficiency among regions had increased, so the spatial pattern had been changing.
3. COVID-19 has affected China’s tourism. With a high degree of marketization, 11 provinces regions had been hit, and the tourism efficiency decreased significantly. Especially in Guangdong and Liaoning, the tourism efficiency had fallen down to the bottom. Because the demand is declining, which leads to the input factors cannot meet the demand. But the tourism efficiency of Guangxi, Zhejiang and Hainan remained stable.

From the changes in the spatial pattern, it can be seen that the tourism efficiency of 11 provinces regions are not similar. If tourism efficiency improves, the gap between regions will narrow. Once the tourism efficiency is reduced, the imbalance between regions will widen.

This paper also draws the spatial distribution of mean MI of 11 provinces regions. The result is shown in Fig 4. According to the numerical size, the mean MI are also divided into five parts. From the perspective of geographical distribution, Guangdong and Jiangsu are centers of 11 provinces regions, with highest MI. Fujian and Shandong, which are neighboring the two provinces, also have a high value. Due to the growth in scale efficiency, the MI of 11 provinces regions is above 1.00, indicating that it is all on an upward trend. Tourism is playing an active role. But we need to pay attention to Guangxi and Hebei because of the low MI.

**Fig 4:** Spatial Differences of MI in 11 coastal provinces regions.

Locations have an impact on tourism. Because tourism has an agglomeration effect, a high level of regional economy will drive tourism efficiency. In order to clarify the difference of tourism efficiency, this paper also divides 11 provinces regions according to the analysis of regional distribution.

The article "Analyzing the tourism efficiency and its influencing factors of China’s coastal provinces" was published in 2024. Journal: PLoS One.

It can be found that the tourism in the Pearl River Delta Economic zone has the highest TE and its value is 0.866. The second one is the Yangtze River Delta Economic zone and its value is 0.865. Finally, the Bohai Economic zone is the lowest and its value is 0.8235 (shown as Table 5). The gap between each other is small and the degree of development is high.

**Table 5:** Tourism efficiency and decomposition for economic zone.

zone	Provincial regions	TE	PE	SE
Pearl River Delta Economic zone	Heibei, Liaoning, Shandong, Tianjin	**0.861**	**0.994**	**0.866**
Yangtze River Delta Economic zone	Jiangsu, Shanghai, Zhejiang	**0.820**	**0.996**	**0.823**
Bohai Economic zone	Fujian, Guangdong, Guangxi, Hainan	**0.863**	**0.997**	**0.865**

It can be drawn from Table 5 that the first one is the Yangtze River Delta Economic Zone. Its tourism infrastructure is well-established, and it also has a high level of urbanization with more abundant, concentrated natural and cultural landscape resources. Meanwhile, the industrial scale advantage of the Yangtze River Delta Economic Zone is obvious. The GDP of the Yangtze River Delta Economic Zone was 20.66 trillion yuan in 2020, accounting for 43.41% of overall 11 coastal provinces regions in China. The Yangtze River Delta Economic Zone has the most abundant resource, with the number of star rated hotels being 1186, accounting for 31.02%; the number of travel agencies was 7759, accounting for 38.39%; the number of A-level scenic spots was 1572, accounting for 28.6%; and the tourism revenue was 1920.9 billion yuan, accounting for 37.86%, the number of tourists was 1277.58 million, accounting for 31.92%.

The second zone is the Pearl River Delta Economic Zone. Its tourism benefits in terms of location, economic foundation, and resident income. The Pearl River Delta Economic Zone has advantages in convenient transportation. It does not only reflect on attracting national travelers, but also foreign travelers, indicating that the area has a large domestic and foreign market. The GDP of the Pearl River Delta Economic Zone had already exceeded 18.24 trillion yuan in 2020. accounting for 34% of overall 11 coastal provinces regions in China. The Pearl River Delta Economic Zone had perfect tourism facilities and resources too, with the number of star rated hotels being 1432, accounting for 37.46%; the number of travel agencies was 6177, accounting for 30.57%; the number of A-level scenic spots was 1567, accounting for 28.5%. and the tourism revenue was 1775.3 billion yuan, accounting for 34.99%. The number of tourists was 325.87 million, accounting for 33.13%.

The article "Analyzing the tourism efficiency and its influencing factors of China’s coastal provinces" was published in 2024. Journal: PLoS One.

The last one is the Bohai Economic Zone. As the birthplace of Chinese culture, it has a long history and the richest in tourism resources among three areas, with the number of A-level scenic spots being 2359 in 2020. At the same time, it is mostly located in plains with superior transportation conditions. There were also 6271 travel agencies and 1205 star-rated hotels, bringing a large number of tourists. Compared to the above two areas, its tourism revenue was only 1376.3 billion yuan in 2020, accounting for 27.13% of overall 11 coastal provinces regions in China.

In summary, the three zones are developed areas and the level of development is approximately the same. But the spatial difference of tourism efficiency is significant, southern areas outperform the northern area. Specific to certain provinces, these 11 coastal provinces regions have spatial differences too. In 2010, the provinces with optimum technical efficiency were only Guangdong and Liaoning. And the overall provincial regions are optimum in 2020, indicating Guangdong and Liaoning are the regions with stable tourism; Shandong, Fujian, Shanghai, Jiangsu, Tianjin and Zhejiang are relatively developed regions with higher technical efficiency; Hainan, Guangxi and Hebei are relatively underdeveloped regions, while these tourism developments are unstable. The proportion of 11 coastal provinces regions for developed, relatively developed and relatively underdeveloped is 2:6:3. The degree of development in 11 coastal provinces regions is mainly concentrated in relatively developed and relatively underdeveloped. Its spatial distribution shows an oval pattern, and there is no obvious spatial correlation.

### 4.4 Coordination analysis

The role of the economy in accelerating tourism is self-evident [59]. To better understand the tourism development in 11 coastal provinces regions, this paper calculates the coordination between tourism efficiency and macroeconomic in these 11 coastal provinces regions by using each provincial GDP growth rate to represent the macroeconomic (shown as Table 6).

**Table 6:** The coordination analysis in 11 coastal provinces regions.

Proj.	2010	2011	2012	2013	2014	2015	2016	2017	2018	2019	2020
Fujian	0.338	0.300	0.283	0.266	0.253	0.231	0.212	0.209	0.211	0.188	0.099
Guangdong	0.296	0.249	0.208	0.213	0.198	0.202	0.190	0.190	0.174	0.160	0.088
Guangxi	0.317	0.312	0.283	0.272	0.230	0.224	0.179	0.196	0.185	0.156	0.109
Hainan	0.401	0.326	0.267	0.263	0.237	0.221	0.190	0.194	0.160	0.151	0.104
Hebei	0.313	0.321	0.286	0.263	0.208	0.205	0.192	0.182	0.173	0.172	0.131
Jiangsu	0.339	0.299	0.276	0.260	0.228	0.224	0.203	0.186	0.173	0.153	0.115
Liaoning	0.251	0.270	0.230	0.225	0.148	0.079	0.014	0.119	0.148	0.141	0.021
Shandong	0.257	0.266	0.239	0.232	0.215	0.204	0.194	0.189	0.163	0.139	0.108
Shanghai	0.309	0.209	0.190	0.205	0.185	0.196	0.178	0.179	0.174	0.156	0.055
Tianjin	0.377	0.355	0.325	0.273	0.209	0.186	0.161	0.096	0.091	0.127	0.042
Zhejiang	0.318	0.251	0.228	0.228	0.223	0.202	0.190	0.197	0.181	0.174	0.091

This is an interesting phenomenon. From the experience of the world, the tourism development trend is consistent with the macroeconomic with the increase in the proportion of the economy. But the results indicate that the tourism development and macroeconomic in 11 coastal provinces regions are not coordinated. There are three reasons: Firstly, the current situation has significant changes. The Chinese economy has been upgrading, and the government pays more attention to reform and quality. As a result, the traditional tourism industry is being replaced by the Internet, and growth is sluggish. At the same time, China and the USA have continuous frictions since 2016, which affects the international economy. Foreign tourism has been greatly impacted. And the COVID-19 has also hit tourism deeply, slowing down the economic recovery. Above all, tourism has affected efficiency. It shows the instability of tourism in 11 provinces’ regions. And, there are also spatial differences in 11 coastal provinces regions. The rapid economic growth in southern areas has promoted the development of tourism, presenting a higher level of coordination.

The article "Analyzing the tourism efficiency and its influencing factors of China’s coastal provinces" was published in 2024. Journal: PLoS One.

From Spatial Differences of the Coordination (shown as Fig 5), it presents a characteristic of "Intermittent sorting" in terms of coordination. Tourism in Fujian has the most coordination. Hebei, Jiangsu, Guangxi and Hainan have also been more coordinated with macroeconomic. As the reforms deepen, the overall area has a slower economic growth rate, which affects tourism development. And the overall provincial regions tend to be consistent. Comparing the mean, the Pearl River Delta Economic Zone with 0.22 is a little higher than the Yangtze River Delta Economic Zone with 0.21. And the Bohai Rim Economic Zone is the lowest with 0.19.

**Fig 5:** Spatial Differences of coordination in 11 coastal provinces regions.

Additionally, there is also a time difference. The tourism development had a higher degree of coordination with the macro economy, that transfers between the southern area and central area from 2010 to 2017. Then, the northern area began to develop into a highly coordinated dispatch system after 2017. At the provincial level, there are different trends: the degree of coordination has been declining in Tianjin, Shanghai, Fujian and Hainan from 2010 to 2020. Guangxi, Guangdong, Hebei and Shandong maintained an increase. Jiangsu, Zhejiang, and Liaoning remain stable, with Jiangsu, Zhejiang is at a high level, while Liaoning is at a low level (shown as Figs 6 and 7).

The article "Analyzing the tourism efficiency and its influencing factors of China’s coastal provinces" was published in 2024. Journal: PLoS One.

**Fig 6:** Spatial Differences of coordination from 2010.

**Fig 7:** Spatial Differences of coordination from 2020.

To sum up, although the regional tourism development gap in 11 coastal provinces regions is narrowed, the overall tourism efficiency shows a trend of differentiation, and the spatial distribution also shows an uneven distribution.

With the central provinces as the core, the spatial coordination in neighboring provincial regions should be expanded to form a tourism concentration zone. The neighboring provincial regions can rely on the proximity advantage, actively develop cross-border tourism and realize the integration of tourism. At the same time, enhancing the convenience of transportation infrastructure and industrial cooperation will help increase the tourism coordination [60].

### 4.5 Driving factors analysis

The driving factors of efficiency mainly include: resources, infrastructure, location, human support, economic, industrial structure, urbanization, informatization, marketization, openness, policy and so on. The factors varied between studies, most scholars focus more on the driving factors of a certain sub-industry. For example, Buhalis observe the main changes in e-Tourism, analyzing the strategic lines that are driving its evolution. He expounded on the significance of linking information and tourism [61]. Figueroa examined Chile as a case study, a country with a growing number of tourists and increased investment in tourist and cultural infrastructures. Empirical results show that cultural endowments and activities together with natural resources determine Chilean regional efficiency in optimizing tourist flow [62]. Using the West Coast of the Strait urban agglomeration, China, as an example, Y Li uses DEA to analyze the nonlinear relationship between tourism economic contact intensity and tourism industry efficiency by constructing a mixed effect model. The result shows that the regional economic level harms the efficiency of the tourism industry. And the urbanization level has a positive effect on the efficiency of the tourism industry [63]. The literature review is shown as Table 7.

**Table 7:** Literature review of driving factors.

Author	Driving Factors
LSY Han (2002)	Natural and/or cultural resources
Buhalis (2008)	Consumers and demand,Technological innovation
Figueroa, (2018)	Cultural endowments and Activities together with natural resources
Y Li et al (2020)	Economic level,Urbanization
M Song, H Li (2019) [64]	Economic development, Urbanization, and The degree of opening up
Alipour. H, Kilic. H (2005) [65]	Internal factors (i.e., institutions)
S. Kytzia, A. Walz, M. Wegmann (2011) [66]	The economic impact of tourists, Occupancy intensity, and The density of beds per area covered by residential buildings and hotels.
Sami Ben Aissa, Mohamed Goaied (2016)	International attraction, Market competition and General tourism wages

Based on the analysis of the literature, this paper selects economic level, consumers and demand, urbanization, general tourism wages and the degree of opening up as the influencing factors to construct the model. (1) Economic level. GDP is an important indicator of the economic development level of a certain province. The high level of economic development can promote the development of tourism. It provides more financial funds for the construction, and also brings more talents, promoting the sustainable development of tourism. So this paper uses GDP as a driving factor of tourism efficiency. (2) Consumers and demand. The consumer demand is an important driver for tourism’s development. With incomes rising, there is more demand for travel, leading to the increase in factor input, the improvement of the industrial sector, and the enriches the tourism experience. (3) Urbanization. Urbanization is the positive factor for promoting the development of the services industry. Urbanization can drive regional economic growth, promote the development of the service industry and enhance the level of marketization. There is also a clear impact on tourism. providing financial, labor, technical and policy support. (4) General tourism wages. Tourism is a labor-intensive industry, and the demand for labor is large. So, labor is an indispensable influencing factor in tourism. Not only the number of labor, but also the quality of labor, the demand for labor in tourism is comprehensive. High-quality labor plays an irreplaceable role in improving efficiency and promoting tourism. General tourism wages can represent the attractiveness of the labor force, and can also reflect the whole picture of tourism. (5) The degree of opening up. The level of opening up is a key factor in the regional economy. As an important part of the service industry, tourism will accelerate its development with the level of opening. The level of opening up plays an important role in the regional economy, and this role will also have an impact on tourism, attracting tourism talent and technology, so as to improve tourism efficiency.

The article "Analyzing the tourism efficiency and its influencing factors of China’s coastal provinces" was published in 2024. Journal: PLoS One.

According to the measurement results of DEA efficiency, the comprehensive technical efficiency is taken as the interpreted variable. And the restricted dependent variables are divided into five parts, including economic level, consumer and demand, urbanization, general tourism wages and the degree of opening up. The overall data is derived from the websites of the National Bureau of Statistics (shown as Table 8).

**Table 8:** Tobit model analysis results.

Variable	Regression Coefficients	Standard error	T	P
economic level	2.543	1.778	4.744	0.000
consumer and demand	4.625	3.313	4.362	0.000
Urbanization	-2.653	0.859	1.995	0.002
general tourism wages	0.555	2.689	-3.106	0.685
the degree of opening up	0.802	0.266	0.532	0.003

Economic level, consumer and demand are positively correlated with tourism efficiency. Among them, consumer and demand have more significant and positive impacts on tourism efficiency than economic level. The development of tourism is a weather vane for a better life [67]. And consumption upgrading of tourism meets the needs for people’s better lives and drives people’s demand in return. As the economic level improves, and residents’ incomes rise, the consumer demand for tourism is the major factor in tourism’s economic vitality. At present, policies targeting the stimulation of tourism consumption have been introduced across China. The demand for tourism is also growing rapidly and the tourism market is sufficient. Now, the government pays more and more attention to tourism, which drives tourism as a “head industry [68]” and gives full play to the huge value of tourism. The importance in the industrial structure has been highlighted. But the degree of opening up only has a slight correlation with tourism efficiency. The reason is that the 11 coastal provinces regions have a high level of opening up, and there is no difference in talent and technology, so the impact cannot be significant.

Urbanization is significantly negatively correlated with tourism efficiency. It can be said that the promotion of urbanization has improved tourism construction with high return, and high returns can absorb more capital investment. But large-scale investment in urbanization may result in excessive waste of tourism resources and flawing in tourism efficiency. To avoid homogenization of tourism, each provincial region should make use of the differences in resources, actively innovate in the period of demand increasing, and improve tourism efficiency.

General tourism wages cannot pass the test. The labor force is the basic driving factor of tourism. This could be that tourism has a large number of employees, but the low level of knowledge of employees has a negative impact on tourism efficiency and general tourism wages are also affected by many factors, which cannot represent the real level of labor force quality, so it is impossible to evaluate efficiency.

The article "Analyzing the tourism efficiency and its influencing factors of China’s coastal provinces" was published in 2024. Journal: PLoS One.

## 5. Conclusion

In this paper, the DEA model is used to measure and analyze the tourism efficiency in 11 coastal provinces regions from 2010 to 2020, and the following conclusions are drawn.

1. This is different from others that the tourism efficiency of 11 provinces regions is not optimistic. As developed regions, the tourism efficiency of 11 provinces regions reached optimal value of 84.68% from 2010 to 2020. Although, it showed a rapid growth trend before 2019. While on the impact of the COVID-19, the scale efficiency declined suddenly and it led to low productivity. This indicates that there is a certain instability in tourism. And the pure technical efficiency in each province stays stable that is closed to the optimal level. The change trend of scale efficiency and comprehensive efficiency is roughly the same. So this paper finds the scale efficiency dominates the value of the efficiency. If the 11 coastal provinces regions expand the tourism scale, the tourism efficiency will be significantly improved.
2. By analyzing the dynamic trend from 2010 to 2020, it is found that the average increase of technical efficiency is 14.0%, the average increase of technical change is 9.5%, and the average increase of MI index is 25.4%. These values remain at a relatively high level. This indicates that tourism of 11 coastal provinces regions has a growing trend and has done relatively well in management and technology. We find that it plays a more important role in driving the growth with the continuous improvement of technology. The reason is that overall 11 coastal provinces regions which are located in a coastal area are able to play the talent effect, and also have advantages in technology application and development.
3. This paper also finds that the spatial difference of tourism efficiency is significant. This means that there are disparities even within developed regions. The overall tourism efficiency of 11 coastal provinces regions in China is on the rise. But due to the differences in conditions, resources, and investment, there is also a significant difference in scale efficiency among them. There is a coordinated relationship between tourism efficiency and macroeconomy, which showed a downward trend from 2010 to 2020. The southern area is better than the northern area. Some provinces such as Guangdong are close to the optimal, while Fujian, Shandong, Liaoning, and Jiangsu also achieve high input-output level. Few provinces have poor performance, especially for Hebei is lowest, its average scale efficiency is only 63.15%, restricting its tourism efficiency. After analyzing the data samples, it was found that there is no obvious spatial correlation, which is shown as an "elliptical" pattern.
4. The most important conclusion distinguishes from others: tourism efficiency is deeply affected by consumer and demand. Economy level, consumer and demand and the level of opening up are positively correlated with tourism efficiency. Consumer demand has a more significant positive impact on tourism efficiency than economy level and the level of opening up. The growth of consumer demand will expand the market scale and improve tourism efficiency. Urbanization has a negative impact on tourism. The promotion of urbanization may result in excessive waste of tourism resources, and the low level of knowledge of employees restricts tourism efficiency.

The article "Analyzing the tourism efficiency and its influencing factors of China’s coastal provinces" was published in 2024. Journal: PLoS One.

Based on the above analysis and empirical results, the following suggestions are proposed:

1. To promote the development of tourism at an appropriate scale. The low scale efficiency restricts the development of 11 coastal provinces’ tourism regions. Therefore, the input of tourism should be expanded, including travel agencies, star-rated hotels and other tourism resources, so as to increase the scale of the tourism. But the 11 coastal provinces regions should rationally adjust input-output resources according to their own conditions in order to avoid homogenization of tourism. Once investment is easily increased, it may result in excessive waste of tourism and restrict tourism development in return.
2. Economic capacity for development should be cultivated, and efforts should be made to raise the income level of residents and provide economic support for the development of tourism. The reason for the regional differences of tourism efficiency in these 11 coastal provinces regions is the unreasonable allocation and utilization of resources. The transformation of tourism is the requirement for high-quality development. Overall, provincial regions should dig deeper into tourism resources, explore more potential of tourism resources, and improve the tourism appeal [69]. This will bring more consumer demands.
3. It is necessary to innovate technological and management. The development of science and technology also contributes a lot to the improvement of tourism efficiency. The 11 coastal provinces regions should improve technological and management with integrate and optimize resources, driving the development of tourism towards innovation. Technology in digitalization, internet, statistics and artificial intelligence should be introduced to effectively improve the management ability and improve the satisfaction of tourists. And the government can better tap into resource potential, draw on various tourism festivals to create multiple distinctive tourism routes and develop targeted tourism creative products based on the connotation characteristics of each tourism resource [70].
4. Accelerating institutional and regional integration, integrating and optimizing resources to promote the deep development of tourism. The tourism industry is open, and it is also a necessary choice to strengthen regional synergy. At present, the tourism market is gradually transitioning to industrial integration. The regional correlation of tourism is strong. Overall, 11 coastal provinces regions that have tourism resources with great local characteristics have advantages in urbanization, transportation, and conditions for tourism integration. They should improve institutional synergy, give support to the integration of tourism, culture, sports, music, and other related industries, and achieve coordination within industrial regions.
